The article "Differential Expression and Bioinformatics Analysis of tRF/tiRNA in Endometriosis Patients" was published in 2022. Journal: Biomed Res Int.

# Differential Expression and Bioinformatics Analysis of tRF/tiRNA in Endometriosis Patients

**DOI:** 10.1155/2022/9911472

**Published:** 2022-03-03

**Authors:** Wang-shu Li, Yi-lin Li, Rui Cao, Chun-fang Ha, Shu Sun, Lan Yu, Jian Li

**Affiliations:** ^1^Department of Gynecology, Dalian Women and Children's Medical Center (Group), 1 Dunhuang Road, Shahekou District, Dalian City, China; ^2^Department of Obstetrics and Gynecology in General Hospital, Key Laboratory of Fertility Preservation and Maintenance of the Ministry of Education, Ningxia Medical University, Yinchuan, Ningxia, China

## Abstract

**Background:**

Endometriosis (EMs) is a benign chronic condition that tends to recur in women of childbearing age, with an incidence of approximately 10%. It is a multifactorial disease for which the pathogenesis is currently unclear. This study is aimed at investigating the expression and clinical significance of tRNA-derived small RNA (tsRNA), a novel noncoding small RNA with potential regulatory functions, in endometriosis.

**Methods:**

The tRF/tiRNA expression profiles in endometrial tissues from three pairs of endometriosis patients and controls were detected by tRF&tiRNA PCR microarray technology and then verified by quantitative real-time polymerase chain reaction (qPCR). The target genes and target sites of TRF396, tiRNA-5030-GlnTTG-3, TRF308, and TRF320 were predicted by miRanda, and the network diagram of their interaction with miRNA was drawn. The impact of tRNA-derived fragments on the pathogenesis of endometriosis was analyzed using the Gene Ontology (GO) and Kyoto Encyclopedia of Genes and Genomes (KEGG).

**Results:**

Two upregulated and 19 downregulated tRNA-derived fragments were identified. The qRT-PCR results of 2 upregulated and 2 downregulated RNA-derived fragments were consistent with the RNA Seq data. The OR2B4 gene related to TRF396, the DGAT1 gene related to tiRNA-5030-GlnTTG-3, the KLF16 gene of TRF308, and the RNF213 gene of TRF320 had significant correlations. Gene Ontology and pathway analysis showed that the target genes of TRF396 and tiRNA-5030-GlnTTG-3 were mainly involved in the intrinsic components of the membrane and the overall composition of the membrane in cell components; molecular functions mainly involve olfactory conduction and G protein-coupled receptor activity. In the biological process, it was mainly involved in the detection of sensory stimuli. The target genes of TRF308 and TRF320 were mainly involved in the intracellular part; molecular functions are mainly related to DNA binding transcription factor activity and protein binding and mainly related to biological regulation of biological processes. Pathway analysis showed that the RAP1 signaling pathway and the AXON GUIDANCE signaling pathway may participate in the progression of endometriosis.

**Conclusion:**

The differential expression of tRF/tiRNA in endometriosis may be related to the pathogenesis of endometriosis. Furthermore, tRF/tiRNA may be a biomarker for the diagnosis and treatment of EMs in the future.

## 1. Introduction

Endometriosis (EMs) is characterized by ectopic growth of endometrial-like tissue outside the uterus [1]. 76% of patients with endometriosis are between 25 and 45 years old, and the typical symptoms of EMs include periodic pelvic pain, dysmenorrhea, dyspareunia, and infertility [2]. The etiology and pathogenesis of EM are still unclear [3]. There is evidence that EMs is a multifactorial disease of which susceptibility factors are suggested as retrograde menstruation, immune system disorders, and genetic and environmental factors [1, 4]. Sampson's retrograde menstruation is now the most widely accepted among all theories of pathogenesis. But there are only 10-15% of women suffering from EMs, while 95% of women experience some degree of menstrual retrograde. Currently, laparoscopic surgery combined with gonadotropin-releasing hormone analogues (GnRHa) is considered to be an effective treatment for endometriosis. However, early diagnosis and treatment of EMs are difficult due to the unclear etiology and nonspecific early symptoms [5, 6]. Therefore, the identification of biomarkers for early diagnosis of endometriosis is the focus of the current research.

Noncoding RNA, as a type of RNA without the function of being translated into proteins, is widely found in organisms and regulates the expression of target genes [7]. It can be used as a new tool to understand biological processes and identify new therapeutic targets [8]. Recent studies have suggested that a large number of small noncoding RNAs are derived from tRNA. The tRNA-derived small RNA (tsRNA) is not a nonfunctional small molecule fragment produced by random cleavage of tRNA but a regulatory noncoding small RNA involved in the pathophysiological process, with precise sequence structure, 5specific expression patterns, and specific biological effect. tsRNA is a small fragment of RNA with specific size generated by specific nucleases, such as Dicer and Angiopoietin (ANG), shearing on the loop of tRNA in a specific cell/tissue or under specific conditions such as stress [9]. There are two main types of tsRNA: one is the stress-inducing RNA (tiRNA) with a length of 28-36 nts, which are produced by specific cleavage on the anticodon loop of mature tRNA; the other, called the tRNA-derived fragment (tRF), is derived from mature or main tRNA and is approximately 14-30 nts in length [10, 11]. These two types of tsRNA can accumulate in different biological processes in several species and possess very different pathways for biogenesis, which are gradually being discovered [10]. A minimum of six types of tRF/tiRNA are known: tRNA-derived fragment 1 (tRF-1), tRF-3, tRF-5, internal tRF (i-tRF), stress-induced tRNA fragment 3 (tiRNA-3), and tiRNA-5, all of which are derived from cutting different locations of the precursor or mature tRNA transcript. tRF/tiRNA is abundant in most organisms and is related to stress responses, cancer, viral infections, and neurological diseases [12]. However, their biological role is still not well understood. Thus, as an important biological regulator, tRF/tiRNA can be used to explain the molecular mechanism of diseases and may be effective diagnostic biomarkers and therapeutic targets [13].

Differentially expressed miRNAs may be potential biomarkers and therapeutic targets for the diagnosis and treatment of endometriosis, as indicated by a growing number of studies [14, 15]. miRNAs influence the process of certain disease development through binding to mRNAs. It is interesting to note that tRF/tiRNA can also affect the occurrence of diseases by regulating the stability of mRNA in a similar manner [16]. Therefore, we hypothesize that the tRF/tiRNA plays a role in the development of endometriosis. However, the expression of tRFs/tiRNA and its potential role in endometriosis have not yet been clarified. In a recent article, the aberrant expression profile of tRFs/tiRNA in ovarian endometriosis indicates that the dysregulated tRNA-derived fragments may be associated with the pathogenesis and the development of ovarian endometriosis [17].

In this study, the expression levels of tRFs/tiRNA in patients with endometriosis were evaluated by using the RNA chip technology and four tRFs/tiRNAs were confirmed by qPCR. Their biological functions were subsequently assessed utilizing bioinformatics to reveal their potential roles in the pathogenesis of endometriosis (Figure 1). These findings may provide a new perspective for elucidating the molecular mechanism of EMs and future treatments.

## 2. Materials and Methods

### 2.1. Patients and Collection of Endometrial Tissues

Endometrial tissues were all eutopic endometrial tissues obtained from ovarian endometriosis patients (25-45 years old) and nonendometriosis patients (25-45 years old). Patients in the EMs group were all diagnosed with endometriosis grades III-IV according to the revised American Society for Reproductive Medicine (r-ASRM) classification of endometriosis and were in the endometrial proliferative phase at the time of tissue collection. All patients had a normal menstrual cycle (21-35 days), and none of them had received gonadotropin-releasing hormone analogs or other hormone medications for at least 6 months before surgery. All the endometrial tissue samples were in the proliferative phase of the menstrual cycle as confirmed by histological diagnosis. The tissue samples were immediately frozen in liquid nitrogen after being taken out of the body and then stored at -80°C for subsequent experiments.

### 2.2. RNA Isolation and Purification

Total RNA was extracted from the endometrial tissues with the TRIzol Reagent (Invitrogen) and further treated with DNase I to remove the contaminating DNA. RNA purification was performed using the RNeasy® MinElute™ Cleanup Kit (Qiagen), followed by the measurement of RNA concentration and purity in NanoDrop® ND-1000. RNA quality control standards are as follows: the ratio of A260/A280 in RNA solution ranges from 1.8 to 2.1, and the total RNA concentration is greater than 40 ng/*μ*L. Moreover, the integrity of RNA was assessed by agarose gel electrophoresis.

### 2.3. tRF&tiRNA Pretreatment and cDNA Synthesis

To further improve the quality of the extracted RNA, the rtStar™ tRF&tiRNA Pretreatment Kit (Arraystar, Rockville, MD, USA) was used to remove small RNAs that would interfere with qPCR. The rtStar™ First-Strand cDNA Synthesis Kit (3′ and 5′ adaptor) (Cat# AS-FS-003, Arraystar, USA) was then used to create a cDNA library of small RNAs, which were subjected to 3′-terminal deacylation, 3′-cP removal, and 5′-P addition, demethylation, ligation of the 3′ adaptors, hybridization of reverse transcription primers, ligation of the 5′ adaptors, and finally reverse transcription into cDNA.

### 2.4. Real-Time Quantitative PCR Amplification

The obtained cDNA was mixed with Arraystar SYBR® Green qPCR Master Mix (ROX+) (AS-MR-006-5, Arraystar) and added to a 384-well plate. The real-time PCR amplification was performed on the ABI 7900 thermal cycler. Then, analyze the obtained dissolution curve.

### 2.5. Target Gene Prediction

Target genes of TRF396, tiRNA-5030-GlnTTG-3, TRF308, and TRF320 were predicted by TargetScan (Release 6.0) and miRanda (v3.3a). Conserved 8mer and 7mer sites with context++ scores less than -0.1 that match the seed region of each tRF were considered effective biological targets. Threshold of structure scores = 140 and free energy = −1.0 were applied in filtering miRanda predicted results. Intersection of TargetScan and miRanda was selected as the final target genes.

### 2.6. Bioinformatics Analysis

The biological functions of differently expressed tRF/tiRNA were revealed by the pathway and process enrichment analysis. The results were conducted through the following ontological sources: Kyoto Encyclopedia of Genes and Genomes (KEGG) approach and Gene Ontology (GO) biological processes. The predicted targets for tRF/tiRNAs were loaded to the database in order to perform GO annotation and pathway search including biological process (BP), cellular component (CC), and molecular function (MF).

Pathway analysis is a functional analysis mapping genes to KEGG pathways. The *p* value indicates the significance of the pathway correlated to the conditions (the recommend *p* value cut-off is 0.05.)

### 2.7. Verification by Quantitative Real-Time PCR (qPCR)

Four pairs of samples were used for qPCR which was performed to confirm the sequencing data. The tRF/tiRNA used for qPCR meets the following criteria: tRF/tiRNA with complete sequence information, fold change > 3.0, *p* value < 0.05; and expression being detectable in all samples. According to these criteria, two upregulated tRF/tiRNA (TRF396 and tiRNA-5030-GlnTTG-3) and two downregulated (TRF320 and TRF308) were selected for qRT-PCR. RNU6-2 was used as a reference. Use the TRIzol reagent to isolate total RNA from endometrial tissue samples. According to the manufacturer's instructions, use the rtStar™ tRF&tiRNA pretreatment Kit (Arraystar, USA) and rtStar First-Strand cDNA Synthesis Kit (3′ and 5′ adaptor) (Arraystar, USA) to reverse transcribed RNA into cDNA. Then, the cDNA was used to perform qPCR. The primers designed for amplification of the tRF transcripts are listed in Table 1.

PCR was performed in a 20 *μ*L reaction volume, including 2 *μ*L cDNA, 10 *μ*L 2x SYBY Green Pro Taq HS Premix, 0.8 *μ*L qPCR Primer Mix, 0.4 *μ*L ROX Reference Dye (20 *μ*M), and 6.8 *μ*L RNase free water. The reaction was predenatured at 95°C for 10 minutes, followed by 40 cycles of amplification at 95°C for 30 seconds, 95°C for 5 seconds, and 60°C for 30 seconds. Triplicate holes were set for all samples and references. The results were calculated by the double standard curve method and displayed as mean ± standard error of mean (SEM).

### 2.8. Data Analysis

The 2^−ΔΔCT^ method was used for analysis. The ΔCT of each pathway-focused gene in each treatment group was first calculated. The method is as follows: ΔCT (group 1) = average CT − average of HK genes′ CT for group 1 array; ΔCT (group 2) = average CT − average of HK genes′ CT for group 2 array; then, the ΔΔCT was calculated for each gene across two PCR arrays (or groups). ΔΔCT = ΔCT (group 2) − ΔCT (group 1). In general, group 1 is the control and group 2 is the experimental group. Finally, the fold change for each gene from group 1 to group 2 was calculated as 2^−ΔΔCT^. Two-tailed Student's *t*-tests were performed, and a *p* value < 0.05 was considered statistically significant.

## 3. Results

### 3.1. Differential Expression of tRF/tiRNA in Patients with Endometriosis

The differences in all tRF/tiRNA expressions in patients with endometriosis are set out in Table 2. Under the conditions of *p* < 0.05, there were 21 tRF/tiRNAs aberrantly expressed in patients with endometriosis: 2 upregulated tRF/tiRNAs and 19 downregulated tRF/tiRNAs (Table 2). Heat map in Figure 2(a) visualizes the expression levels of 21 differentially expressed tRF/tiRNAs in ovarian endometriosis patients and healthy individuals. The volcano and scatter plots highlighted the changes in tRF/tiRNA expression between the two groups (Figures 2(b) and 2(c)). Among the top 20 tRF/tiRNAs, the expression levels of TRF396 and tiRNA-5030-GlnTTG-3 in the eutopic endometrial tissue of endometriosis patients were higher than those in controls (*p* < 0.05, statistically significant) (Figure 2(d)). The downregulated are TRF320, TRF308, 1042, 1030, and 5008C.

### 3.2. qPCR Verification

To verify the sequencing data, qPCR was performed to confirm the expression changes of two upregulated and two downregulated tRF/tiRNAs. The result revealed that, in the eutopic endometrium of patients with endometriosis, TRF308 was underexpressed while TRF396 and tiRNA-5030-GlnTTG-3 were overexpressed (Figure 3). This is consistent with the results obtained by the tRF&tiRNA PCR chip technology. Although TRF320 and tiRNA-5030-GlnTTG-3 were upregulated in the eutopic endometrium of patients with endometriosis, but they were not statistically significant (*p* > 0.05). In contrast, TRF308 and TRF396 were downregulated by 3.10-fold or upregulated by 1.94-fold, respectively (*p* < 0.05).

### 3.3. Target Gene Prediction

At present, the mechanism underlying the role of tRF/tiRNA in EMs is not yet clear, but there is some evidence indicating that tRF/tiRNAs have similar functions to miRNA. tRF/tiRNAs regulate its stability by binding to mRNA, thereby inhibiting translation, regulating gene expression, cell cycle, and chromatin. Various mechanisms such as epigenetic modification play a biological role [18].

We used miRanda to predict the target genes and target sites of TRF396, tiRNA-5030-GlnTTG-3, TRF308, and TRF320 (Figure 4). GO and KEGG analysis further explained the functions of these genes and their roles in signaling pathways. The analysis led to the results that TRF396, tiRNA-5030-GlnTTG-3, TRF308, and TRF320 are closely associated with OR2B4, DGAT1, KLF16, and RNF213, respectively (Figures 5(a)–5(d)).

### 3.4. GO Enrichment Analysis and Pathway Analysis

The bioinformatics of tRF/tiRNAs was analyzed for understanding their biological functions. The KEGG pathway and the GO biological process were investigated to explore the function of tRF/tiRNAs in endometriosis. The ontology includes three areas: molecular function (MF), cell composition (CC), and biological process (BP).

Visualize the GO analysis of up/downregulated tRF/tiRNA in patients with endometriosis through the bar graph formed by the aggregation of molecular functions, cellular components, and biological processes. The molecular functions of the upregulated tRF/tiRNA mainly involve olfactory transmission and G protein-coupled receptor activity, which mainly participates in the intrinsic components of the membrane and the overall composition of the membrane in cell components and the stimulation of sensory perception in biological processes (Figure 6(a)).

The molecular functions of downregulated tRF/tiRNA mainly involve DNA-binding transcription factor activity and protein binding, which mainly participates in the intracellular part of cell components and biological regulation in biological processes (Figure 6(b)). Functional analysis of four validated tRF/tiRNAs to visualize tRF/tiRNAs pathway enrichment in endometriosis on bar graphs (Figures 7(a) and 7(b)).

## 4. Discussion

The etiology and pathogenesis of endometriosis are still poorly understood. Current surgical procedures and medical treatments for endometriosis are ineffective for the majority of women. Even if the treatments are effective, it is often accompanied by severe complications and a high recurrence rate [19]. Moreover, hormone therapy is not suitable for women with endometriosis who intend to have children [20]. Therefore, in order to develop targeted treatments, it is necessary to have a deeper understanding of the pathogenesis of endometriosis at macroscopic and molecular levels [21].

In recent years, technologies such as noninvasive biomarkers, proteomics, genomics, and miRNA chips are emerging and may contribute to the diagnosis of diseases. These latest techniques can be used to study the complete molecular or genetic profiles of EMs and further evolve into the gold standard diagnostic tool, thereby eliminating invasive laparoscopy [22]. A growing body of evidence demonstrates that ncRNAs, including miRNAs and long ncRNAs, play an important regulatory role in the pathogenesis and development of endometriosis [22, 23]. For example, the overexpression of microRNA-142-3p inhibits the proliferation and the transfer of endometrial cells and the formation of vascular endothelial cell tubes. MicroRNA-142-3p directly targets KLF9 to regulate the expression of VEGFA resulting in the promotion of ectopic endometriotic lesion growth [24]. A study of 104 ectopic endometrial samples from endometriosis patients and 50 normal endometrium samples from controls revealed that the expression of lncRNA H19 in the ectopic endometrium of patients with endometriosis was significantly higher than that in the normal endometrium. It has also been suggested that the overexpression of lncRNA H19 was an independent prognostic factor and the level of lncRNA H19 can predict recurrence through sensitivity and specificity, implying that lncRNA H19 can be used as a predictor of endometriosis recurrence [25]. In endometriosis, transcriptome profile analysis of tissue samples as well as functional studies *in vivo* and *in vitro* has shown that ncRNAs are pivotal factors in the development of the disease [23]. Among them, the small RNA (tsRNA) derived from tRNAs has gradually become well known. Compared with miRNAs and long ncRNAs, tRF/tiRNAs possess a certain degree of tissue specificity and temporal specificity. Studies have proven that the relative abundance of tRF/tiRNA expressed in different tissues and at different periods in the same tissue is specific [26, 27]. Furthermore, tRF/tiRNA not only has the advantage of being detectable in blood and body fluids, but its unique structure and modifications make it more stable and less degradable in the human body [18, 28]. It has been reported that tRF/tiRNA plays a key role in tumorigenesis and some tRFs have the activity to suppress tumors and inhibit their metastasis [29]. In particular in high-grade serous ovarian cancer (HGSOC), tRF-03357 may promote cell proliferation, migration, and invasion by regulating HMBOX1 [30]. Considering that endometriosis has cancer-like features such as adhesion, invasion, neovascularization, and the ability to inhibit apoptosis, the potential role of tsRNA in endometriosis is increasingly being discovered [31].

We found that the tRF/tiRNAs were aberrantly expressed in patients with ovarian endometriosis compared to the control group. The tRF/tiRNAs were differentially expressed in the samples, and tRF/tiRNA may be a candidate for the pathogenesis of ovarian endometriosis. This study verified two upregulated and two downregulated tRF/tiRNAs by qPCR, which were consistent with the tRF/tiRNA sequence data and reflected the expression trend. GO analysis showed that the target genes of TRF396 and tiRNA-5030-GlnTTG-3 are mainly involved in the intrinsic components of the membrane and the overall composition of the membrane in cell components; molecular functions mainly involve olfactory conduction and G protein-coupled receptor activity. The process mainly participates in the detection of stimuli involving sensory perception in biology. The target genes of TRF308 and TRF320 are mainly involved in the intracellular part and molecular functions mainly concerned with DNA binding transcription factor activity and protein binding, mainly involved in biological regulation of biological processes. Recently, the molecular biocharacteristics of the eutopic endometrium have been considered to play an important role in the occurrence and development of endometriosis, and the underlying cause of which may be the difference in gene expression [32]. The “unified” theory of “reign endometrial determinism” put forward by Academician Lang Jinghe believes that the biological characteristics of the reign endometrium of patients with endometriosis lead to the determinants of the disease. The eutopic endometrium of patients with endometriosis has stronger adhesion, invasion, and angiogenesis, which makes endometriosis different from other diseases. In the present study, tRF/tiRNAs were differentially expressed in the eutopic endometrium of patients with endometriosis, indirectly proving that the dysfunction of the eutopic endometrium plays a role in the development of endometriosis.

tRF/tiRNAs primarily play a role in posttranscriptional gene regulation. First, tRF/tiRNA can affect protein translation by competitively binding to the translation initiation complex [33]. tRF and tiRNA may bind to RNA-binding proteins such as Y-box binding protein 1 (YBX1) and block transcription, inactivate the initiation factor eIF4G/A, promote ribosomal protein translation, or activate Aurora kinase A (regulator) [8]. For example, the untranslated region (UTR) of the TRF binding protein YBX1 can inhibit the growth of cancer cells caused by serum starvation, cancer cell invasion, and breast cancer metastasis [34]. Second, tRF/tiRNAs can also be genetically involved in the regulation of DNA damage in a similar manner to miRNAs. A study using miRBase to classify miRNAs that overlap with the sequences of tRFs identified 20 tRNA-derived miRNAs that share sequences with tRFs, with 5 miRNAs (miR-3182, miR-4521, miR-1260a, miR-1260b, and miR-7977) featuring significant prediction scores [16]. It was also discovered that tRF can be loaded onto the Argonaute (AGO) family proteins for posttranscriptional regulation. For instance, Dicer-independent tRF-3, which is produced at the time of tRNA overexpression, can suppress the gene posttranscriptionally via binding to RISC-containing Argonaute-GW182 that matches the target mRNA sequence [35]. The systematic analysis of the Argonaute CLIP-seq dataset also demonstrated that tRF can regulate the posttranscriptional process through a large number of tRF-target gene interactions (TGI) [36]. Argonautes (AGO) are important core proteins in the RNA interference (RNAi) pathway of eukaryotic cells. There are mainly four AGO members (AGO1-4) in humans, which are expressed in cells and tissues [37]. In human cells, tRF is associated with Argonaute 1, 3, and 4, but not with Argonaute 2. Argonaute 2 is the key effector protein of miRNA function but has similar characteristics to miRNA, indicating that tRF may play a major role in RNA silencing [38].

We speculate that the disturbed expression of TRF396 may further regulate the disease process of endometriosis by binding to mRNA as miRNA or by associating with AGO during the occurrence and development of endometriosis. The development of endometriosis involves the interaction of endocrine, immune, proinflammatory, and proangiogenic processes [39]. There is evidence that a number of factors associated with angiogenesis, which plays an essential role in the occurrence and development of endometriosis, are indispensable in endometriosis [22]. Olfactory transduction and RAP1 signaling pathway are closely connected to the dysregulation of tRF/tiRNA (Figure 7(a)). By predicting the target genes of TRF396, we found that it was closely linked to OR2B6 in olfactory receptors (ORs). ORs are expressed in a variety of human tissues and contribute to different physiological processes. Ectopic ORs are implicated in the proliferation, apoptosis, metastasis, and invasive process of tumor cells and take part in the angiogenesis and wound healing process [40]. Among ORs that have been established as biomarkers for certain cancers, OR2W3 and OR2B6 may be tied to the progression of invasive breast cancer [41]. Therefore, the combination of TRF396 and the gene OR2B6 may be a contributor to the pathogenesis of endometriosis, which provides a direction for future research.

RAS-associated protein 1 (RAP1), a member of the small G protein family of RAS, influences the tumor development and progression by engaging in various biological processes such as cell proliferation, invasion, migration, and apoptosis imbalance [42, 43]. A recent study showed that PP2Ac nitration during cAMP-induced decidualization of hESCs was induced through the Epac1-Rap1-PLC*ε*-CaMKII-HDAC5-iNOS signaling pathway [44]. It has been found that RAP1A and EPAC1 were highly expressed in ovarian endometriosis and their expressions were positively correlated, speculating that RAP1A and EPAC1 may cooperate with each other to participate in the occurrence and development of EMs and in the regulation of dysmenorrhea. The MAPK signaling pathway is in the regulation of cell growth and invasion [45]. The RAP1 signaling pathway further acts on the MAPK signaling pathway together engaging in the development of endometriosis (Figures 8(a) and 8(b)). Recently, it has been confirmed that ncRNA regulates ESC through p38 MAPK and PKA/SERCA signal transduction by interacting with Galectin-1. This novel regulatory mechanism can provide new insights for drug treatment and diagnosis of endometriosis [46]. At the molecular level, the activation of p38 MAPK and p42/44 ERK, important regulators of endothelial migration and proliferation, was reduced in Rap1b-deficient endothelial cells [47]. This sheds light on a novel role of RAP1 in the signaling pathway regulating endothelial cells to promote angiogenesis. There is an increasing interest in exploring the function of RAP1 in the proliferation, invasion, adhesion, and neovascularization of eutopic and ectopic endometrial cells in endometriosis, as well as the regulation of cell autophagy to participate in the occurrence and development of dysmenorrhea. The important role of RAP1 in endometriosis further confirmed the important role of tRF/tiRNA in endometriosis. The role of the AXON GUIDANCE/MAPK signaling pathway in endometriosis deserves further exploration (Figures 9(a) and 9(b)).

## 5. Conclusion

Overall, this study revealed changes in the expression of tRF/tiRNA in patients with endometriosis. tRF/tiRNA may be a new potential diagnostic and therapeutic target for endometriosis. Furthermore, due to the multifactorial nature of endometriosis, it would be preferable to use a set of tsRNA biomarkers rather than a single biomarker to improve predictive power and diagnostic accuracy. This research provides the basis and direction for further research. However, this study is limited by the sample size. It would be better to have a larger sample size and clinical specimens to back up the results. The mechanism of tRF/tiRNA action in endometriosis needs to be clarified through more research.

## Figures and Tables

**Figure 1:** Study design illustration.

**Figure 2:** Analysis of differential expression of tRF/tiRNA in patients with endometriosis compared with healthy controls. The heat map depicts 21 differentially expressed tRF/tiRNA in all 6 samples. Control groups 1, 2, and 3 refer to samples from healthy people (*n* = 3); endometriosis 1, 2, and 3 refer to samples from patients with endometriosis diagnosed by laparoscopy (*n* = 3) (a). The volcano and scatter plots show the changes in tRF/tiRNA expression between the two samples (b, c). In patients with endometriosis, the top 20 upregulated/downregulated tRF/tiRNA expressions (d, e).

**Figure 3:** The PCR verification results of four dysregulated tRFs/tiRNA in endometriosis and control groups. Use Student's *t*-test to analyze all data. ∗ indicates a significant difference between the two groups (^∗^*p* < 0.05).

**Figure 4:** Putative genes with context less than -0.4.

**Figure 5:** A DTRF320-related RNF213 gene (Seqname: NM_020954). (a) TRF396-related OR2B4 gene (Seqname: NM_012367). (b) tiRNA-5030-GlnTTG-3-related DGAT1 gene (Seqname: NM_012079). (c) TRF308-related KLF16 gene (Seqname: NM_031918). (d) TRF320 related RNF213 gene (Seqname: NM_020954).

**Figure 6:** (a) The GO analysis of upregulated tRF/tiRNA in patients with endometriosis through a bar graph aggregated by molecular functions, cellular components, and biological processes. b) The bar graph of downregulated tRF/tiRNA through molecular functions, cellular components, and biological processes to visualize the GO analysis of downregulated tRF/tiRNA in patients with endometriosis.

**Figure 7:** (a) The upregulated tRF/tiRNA pathway enrichment in endometriosis on the bar graph. The data shows that these genes are mainly involved in olfactory conduction, carbon metabolism in cancer, complement and coagulation cascade, Rap1 signaling pathway, and other biological processes. (b) The enrichment of the downregulated tRF/tiRNA pathway in patients with endometriosis. The data shows that these genes are mainly involved in cell aging, glioma, and the role of proteoglycans in cancer. Process (the vertical axis shows the annotation function of the target gene. The horizontal axis shows the enrichment score (-log10-converted *p* value) and the number of genes in each cluster, respectively. Only the first 10 significantly enriched clusters are included).

**Figure 8:** (a) Signal pathway prediction. Collect the Kyoto Encyclopedia of Genes and Genomes (KEGG) pathway analysis that expresses upregulated genes (the vertical axis shows the annotation function of the gene. The horizontal axis represents the enrichment score (-log10-converted *p* value) and gene number of each cluster, respectively. Only the most significantly enriched clusters are included). For genes whose expression is upregulated, pathway analysis shows that 15 pathways may be involved, and the figure shows the ten most important pathways. (b) The RAP1 signaling pathway expressing upregulation of MAPK may play an important role in the pathogenesis and progression of endometriosis.

**Figure 9:** (a) The predicted signaling pathways of downregulated expression. Collect the Kyoto Encyclopedia of Gene and Genome (KEGG) pathway analysis of downregulated genes (the vertical axis shows the annotation function of the gene. The horizontal axis represents the enrichment score (-log10-converted *p* value) and gene number of each cluster, respectively). Only the most significantly enriched clusters are included. For genes whose expression is downregulated, pathway analysis revealed that 27 pathways may be involved, and the figure shows the ten most important pathways. (b) The MAPK signaling pathway that downregulates AXON GUIDANCE may play an important role in the pathogenesis and progression of endometriosis.

**Table 1:** tRF sequence.

tRF&tiRNA name	tRF sequence	Source tRNA
tiRNA-5030-GlnTTG-3	GGTCCCGTGGTGTAATGGTTAGCACTCTGG	GlnTTG
TRF396	GGGGGTATAGCTCAGCGGT	AlaAGC
TRF320	GCCGTGATCGTATAGTGGTTA	HisGTG
TRF308	GCCCGACTACCTCAGTCGG	LysCTT

**Table 2:** Under the conditions of *p* < 0.05, compared with the control group, there were a total of 18 tRF/tiRNA differential expressions in the experimental group samples, of which 2 tRF/tiRNAs were upregulated and 16 were downregulated.

		AVG ΔCt (Ct(GOI) − Ave Ct (HKG))		2^−ΔCt^		Fold difference	*t*-test	Fold up- or Downregulation	
Transcript name	Well	Test	Control	Test	Control	Test/control	*p* value	Test/control	Comments
3′tiR_012_ArgCCT (n)	A02|B02	12.90	11.88	0.0001305622	0.0002651040	0.49	0.0217	-2.03	OKAY
3′tiR_026_GlnCTG (n)	A03|B03	11.50	10.72	0.0003449815	0.0005910585	0.58	0.0033	-1.71	OKAY
3′tiR_056_ValTAC (mt)	A06|B06	7.65	6.25	0.0049731201	0.0131295495	0.38	0.0281	-2.64	OKAY
3′tiR_078_ArgTCT (n)	A10|B10	7.65	7.00	0.0049754532	0.0078167154	0.64	0.0384	-1.57	OKAY
5008C	A15|B15	10.77	8.90	0.0005734410	0.0020932464	0.27	0.0445	-3.65	OKAY
5016C	A17|B17	16.50	15.16	0.0000108028	0.0000273061	0.40	0.0389	-2.53	B
TRF419	A23|B23	13.85	12.21	0.0000676452	0.0002109906	0.32	0.0439	-3.12	B
tiRNA-5033-ProTGG-1	A24|B24	7.94	7.04	0.0040641490	0.0076003464	0.53	0.0018	-1.87	OKAY
tiRNA-5031-PheGAA	C17|D17	10.47	9.68	0.0007030109	0.0012169640	0.58	0.0382	-1.73	OKAY
tiRNA-5030-GlnTTG-3	C19|D19	16.60	18.34	0.0000100786	0.0000030114	3.35	0.0403	3.35	OKAY
1001	E08|F08	19.05	17.23	0.0000018452	0.0000065217	0.28	0.0478	-3.53	B
1030	E24|F24	18.85	16.97	0.0000021147	0.0000078082	0.27	0.0009	-3.69	B
1035	G04|H04	19.82	18.15	0.0000010836	0.0000034430	0.31	0.0204	-3.18	C
1042	G11|H11	19.21	16.81	0.0000016479	0.0000087138	0.19	0.0016	-5.29	B
3033A	G16|H16	10.14	9.42	0.0008843119	0.0014609092	0.61	0.0407	-1.65	OKAY
3006A	G22|H22	11.76	10.52	0.0002879253	0.0006802099	0.42	0.0109	-2.36	OKAY
3008B	G24|H24	19.30	17.56	0.0000015512	0.0000051712	0.30	0.0362	-3.33	OKAY
3011/12A	I02|J02	6.64	6.21	0.0100170904	0.0135292833	0.74	0.0050	-1.35	OKAY
TRF308	M06|N06	17.47	15.57	0.0000055225	0.0000206195	0.27	0.0306	-3.73	C
TRF320	M10|N10	18.89	16.82	0.0000020591	0.0000086166	0.24	0.0177	-4.18	C
TRF396	O02|P02	14.01	16.51	0.0000607708	0.0000107517	5.65	0.0070	5.65	C

“OKAY”: the average Ct is relatively high (>30) in one of the samples but is still relatively low in the other sample (<30), suggesting that the fold change value may not be as accurately calculated. “B”: the average Ct values are relatively high (>30) in both control and test samples, and the *p* value is either unavailable or above cut-off (*p* > 0.05). More biological replicates are needed to detect differential expression at low expression levels. “C”: the average Ct values are not determined or greater than the cut-off (default 35) in both samples, indicating that the gene expression is undetected.

## Data Availability

The datasets used or analyzed during the current study are available from the corresponding author on reasonable request.
